The article "A randomized phase II clinical trial of nab-paclitaxel and carboplatin compared with gemcitabine and carboplatin as first-line therapy in locally advanced or metastatic squamous cell carcinoma of lung" was published in 2014. Journal: BMC Cancer.

# A randomized phase II clinical trial of nab-paclitaxel and carboplatin compared with gemcitabine and carboplatin as first-line therapy in locally advanced or metastatic squamous cell carcinoma of lung

**DOI:** 10.1186/1471-2407-14-684

**Published:** 2014-09-20

**Authors:** Jin-Ji Yang, Cheng Huang, Gong-Yan Chen, Yong Song, Ying Cheng, Hong-Hong Yan, Qing Zhou, Yi-Long Wu

**Affiliations:** Guangdong Lung Cancer Institute, Guangdong General Hospital & Guangdong Academy of Medical Sciences, 106 Zhong Shan Dong Er road, Guangzhou, China; Fujian Province Cancer Hospital, 91 Fu Ma road, Fuzhou, China; Heilongjiang Province Cancer Hospital, 150 Ha Ping road, Harbin, China; Nanjing General Hospital, 305 Zhong Shan Dong road, Nanjing, China; Jilin Province Cancer Hospital, 1018 Hu Guang road, Changchun, China

**Keywords:** Nab-paclitaxel, Carboplatin, Gemcitabine, Squamous, Carcinoma, Lung

## Abstract

**Background:**

Recent advances have shown that histology and genetic biomarkers are important in patient selection, which have led to significantly better outcomes for lung cancer patients. However, most new treatments only apply to adenocarcinoma or non-squamous, and in squamous carcinoma there is little breakthrough. In a phase III trial nab-paclitaxel plus carboplatin showed superior response rate over paclitaxel and carboplatin. In subgroup analysis the squamous histology appeared to be a predictive factor to nab-paclitaxel treatment.

**Methods/Design:**

This is an open-label, randomized, active controlled phase II trial. A total of 120 untreated advanced squamous lung cancer patients are randomized at a 1:1 ratio to receive nab-paclitaxel (135 mg/m^2^, d1, 8, q3w) plus carboplatin (AUC 5, d1, q3w) or gemcitabine (1,250 mg/m^2^, d1, 8, q3w) and carboplatin (AUC 5, d1, q3w). The primary endpoint is objective response rate and the second endpoints are progression free survival, overall survival, safety and biomarkers associated with nab-paclitaxel. The treatment will continue up to six cycles or intolerable toxicity.

**Discussion:**

This ongoing trial will be the first prospective randomized trial to explore the efficacy of nab-paclitaxel as the first-line treatment specifically in squamous carcinoma of lung.

**Study number:**

CTONG1002

**Trial Registration:**

Clinicaltrials.gov reference: NCT01236716

## Background

For both men and women, lung cancer is the leading cause of death and non-small cell lung cancer (NSCLC) represents more than 80% of all lung cancer cases [1]. Compared with best supportive care, platinum-based doublet chemotherapy not only prolongs the survival, but also improves symptom control and the quality of life. It has been the standard of care for advanced NSCLC [2]. Available data suggest that different platinum/third generation chemotherapy agent combinations have similar efficacy in the first line setting [3].

The article "A randomized phase II clinical trial of nab-paclitaxel and carboplatin compared with gemcitabine and carboplatin as first-line therapy in locally advanced or metastatic squamous cell carcinoma of lung" was published in 2014. Journal: BMC Cancer.

Traditionally, the choice of chemotherapy is based on performance status, age, etc, and histology has not influenced the treatment options. Recent years, personalized treatment has developed rapidly with the emerging of new chemotherapy agents and targeted therapies. Pemetrexed has favorable efficacy and safety profiles in non-squamous NSCLC but not in squamous population [4]. The benefit of bevacizumab is also limited to the non-squamous subtypes [5]. Moreover, most targeted drugs need molecular markers to distinguish patients who would likely to gain survival advantage from treatment, such as epidermal growth factor receptor (EGFR) mutation for EGFR tyrosine kinase inhibitors (TKIs) [6, 7], EGFR amplification for cetuximab [8] and anaplastic lymphoma kinase (ALK) fusion-positive for ALK inhibitor crizotinib [9]. Molecular-targeted drugs have the advantages of prominent therapeutic efficacy and moderate adverse reactions, prolonging patients’ survival time and improving the quality of life at the same time. EGFR-TKIs such as erlotinib and gefitinib have been recommended as the first -line treatment in EGFR mutation patients by clinical practice guidelines [2].

Despite all the progress in adenocarcinoma and biomarker positive patients, the treatment breakthroughs for squamous histology are few. Although the EGFR mutated squamous lung cancer patients can be treated with EGFR-TKIs as well, the mutation rate in this population is much lower than that in the non-squamous subtypes (around 10% in Caucasian adenocarcinoma patients, 30% in Asian adenocarcinoma patients, but only around 3% in squamous patients [10]). Thus major part of squamous patients remains on platinum-based doublet with an average objective response rate (ORR) around 20% and overall survival (OS) no longer than 12 months.

Nab-paclitaxel (Abraxane) is a nano-technology developed albumin bound paclitaxel. With the natural affinity of albumin to tumor cells, it enables paclitaxel to be concentrated in cancer lesion to exert bigger anti-neoplastic effect. In a phase III trial of Abraxane plus carboplatin versus solvent-based paclitaxel [11], Abraxane arm shows significantly higher ORR than the solvent-based paclitaxel arm (33% vs 25%, p = 0.005) and equivalent progression free survival (PFS) and OS. The ORR benefit is especially bigger in squamous subtype (41% vs 24%, p < 0.001) and the OS beneficial trend is bigger in this group too.

With these promising findings of subtype analysis in the phase III trial, this trial is designed to prospectively explore the efficacy of Abraxane specifically in the squamous population by a head to head comparison to current standard of care.

The article "A randomized phase II clinical trial of nab-paclitaxel and carboplatin compared with gemcitabine and carboplatin as first-line therapy in locally advanced or metastatic squamous cell carcinoma of lung" was published in 2014. Journal: BMC Cancer.

## Methods/Design

This study is a multicenter, randomized, active controlled, open label phase II clinical trial. The objective is to study the efficacy and safety of nab-paclitaxel and carboplatin compared with gemcitabine and carboplatin as first-line therapy in advanced squamous cell carcinoma of lung. All patients in this study have locally advanced or metastatic squamous cell carcinoma of lung which has been histologically confirmed. The inclusion and exclusion criteria are summarized in Table 1. This study was approved by the ethics committees of Guangdong General Hospital, Fujian Province Cancer Hospital, Heilongjiang Province Cancer Hospital, Nanjing General Hospital and Jilin Province Cancer Hospital respectively.Recruitment for this study is currently ongoing in 5 sites in China. Written informed consent must be provided by all patients before any trial-related procedures are carried out. 120 patients are randomly assigned to treatment group A: receiving nab-paclitaxel 135 mg/m^2^, d1, 8 and carboplatin AUC 5, d1 every three weeks; or group B: receiving gemcitabine 1,250 mg/m^2^, plus carboplatin AUC 5, d1 every three weeks. Both group A and B receive up to six cycles of chemotherapy.

**Table 1:** **Inclusion and exclusion criteria**

**Inclusion criteria**	• Previously untreated, histologically documented stage IIIB to stage IV or stage IIIA that is not amenable to regional therapy (7^th^ Edition of TNM Staging Criteria) squamous cell carcinoma of lung. Previously untreated, histologically documented squamous cell carcinoma of lung with stage IV or locally advanced disease that is not amenable to radical regional therapy (7^th^ Edition of TNM Staging Criteria).
	• At least one measurable tumor lesion as defined by RECIST criteria.
	• 18 to 85 years of age.
	• ECOG performance status 0-1.
	• Patients have no previously malignant tumors or history except cured cervical carcinoma in situ, basal cell carcinoma or superficial bladder cancer (T_a_, T_is_ or T_1_).
	• Patients should not have been treated with chemotherapy such as gemcitabine, platinum and taxane. But patients who have received chemotherapy for neoadjuvant or adjuvant treatment at least 12 months before the study treatment are eligible.
	• Patients’ blood test must meet the following requirements:
	o ANC ≥ 1.5 x 10^9^/L
	o Platelets ≥ 100 x 10^9^/L
	o Hb ≥ 90 g/L (9 g/dL)
	• Patients’ clinical biochemistry examination must meet the following requirements:
	o ALT and AST ≤ 2.5 x upper limit of normal (ULN) without liver metastasis, ALT and AST ≤ 5 x ULN with liver metastases
	o Serum creatinine ≤ 1.5 x ULN
	o Total bilirubin ≤ 1.5 x ULN
	• Urine pregnancy test is negative for women, within 14 days before study treatment.
	• Estimated life expectancy of at least 3 months.
	• Patients will comply with the clinical trial protocol.
	• Patients voluntarily participate in clinical trial and the informed consent must be signed.
**Exclusion criteria**	• Patients who are currently undergoing other anti-tumor therapies.
	• Patients who were enrolled into any other clinical trial within 4 weeks of study entry.
	• Any clinical laboratory findings give reasonable suspicion of a disease or condition that contraindicates the use of any study medication or render the subject at high risk from treatment.
	• Primary brain tumor or central nervous system metastatic tumor.
	• Serious mental disorder.
	• Serious dysgnosia or cognitive dysfunction.
	• Other serious comorbidities.
	• Alcohol or drug dependence.
	• Previously allergic to drugs used in the study.
	• Patients who are deemed unsuitable to participate in the study

The article "A randomized phase II clinical trial of nab-paclitaxel and carboplatin compared with gemcitabine and carboplatin as first-line therapy in locally advanced or metastatic squamous cell carcinoma of lung" was published in 2014. Journal: BMC Cancer.

### Study objectives

The primary objective of this study is to compare the ORR of Abraxane plus carboplatin to gemcitabine plus carboplatin. Secondary objectives include PFS, OS, safety and biomarker parameters. Exploratory endpoints include expression of secreted protein acid rich in cysteine (SPARC) and caveolin-1 in NSCLC tissue and their predictive value in PFS and OS. Tumor samples will be collected from all randomized patients and tested in the central lab of Guangdong Lung Cancer Institute, Guangdong Academy of Medical Sciences.

### Statistics

The sample size calculation assumes that in advanced squamous lung cancer, Abraxane + carboplatin has an ORR of 40% [11] while gemcitabine + carboplatin has an ORR of 19% [3]. With inequality test using ratios of two independent proportions, the sample size is 120 patients in total, which will be randomly assigned at a 1:1 ratio between two treatment arms (60 in each). This sample size will provide 80% power with two-sided type I error of 0.05 to reject the primary efficacy null hypothesis that Abraxane + carboplatin/gemcitabine + carboplatin hazard ratio for ORR is equal to 1.0.

The primary objective will be analyzed by chi-square test. Secondary endpoints of PFS and OS will be evaluated by Kaplan-Meier method with a 95% confidence interval. The log-rank method will be used to compare the difference between the survival curves of two arms. Multifactorial Cox regression analysis will be used to determine the prognostic factors of the survivals including PFS and OS.

### Ethical considerations

Prior to initiation of the study, each of the participating sites must obtain local or central ethics committee approval from the appropriate body. All research will conform to the Declaration of Helsinki, as well as local legal and ethical requirements.

The article "A randomized phase II clinical trial of nab-paclitaxel and carboplatin compared with gemcitabine and carboplatin as first-line therapy in locally advanced or metastatic squamous cell carcinoma of lung" was published in 2014. Journal: BMC Cancer.

## Discussion

Previous researches have shown comparable efficacy and good safety profile of Abraxane-based chemotherapy in the first-line treatment of advanced NSCLC, compared to other standard platinum-based doublets. In a phase III trial, the ORR of Abraxane plus carboplatin is significantly higher than solvent-based paclitaxel and the survival time is equivalent in two groups [11]. The most common adverse events of interest in Abraxane arm are hematological toxicity and neuropathy. The incidence of Grade 3-4 thrombocytopenia and anemia are higher in Abraxane group than solvent-based paclitaxel arm, while the incidence of neutropenia is higher in solvent-based paclitaxel arm. Generally, the majority of hematological toxicities in both arms are Grade 1-2 and manageable. Grade 3-4 sensory neuropathy occurred more frequently in solvent-based paclitaxel arm than Abraxane arm (12% vs 3%) and the median time to improvement of Grade 3-4 neuropathy to Grade 1 is much less for Abraxane arm than solvent-based paclitaxel arm (38 days vs 104 days). Thus Abraxane seems an optimal choice of third generation chemotherapy agents to be combined with platinum as the standard treatment due to its high activity and favorable safety profile.

Moreover, retrospective subgroup analyses showed that in squamous histology group, there were more significant ORR benefit and OS improvement trend. Squamous cell carcinoma consists approximately 30% of all NSCLC but new treatment options are few. There is huge unmet medical need to increase the prognosis of this patient population. Abraxane has the active agent of paclitaxel, which is an approved agent for treatment of squamous cell lung cancer, as well as the albumin-bound property which increases the drug distribution and concentration to a new level. Furthermore, studies have showed that SPARC is an albumin-bound protein that is rich in tumor matrix and may plays an important role in absorbing Abraxane into the tumor site [12]. SPARC may serve as a predictive or prognostic biomarker of Abraxane-based therapy. Thus Abraxane has the potential to be the optimal treatment choice in squamous carcinoma of lung to achieve better response and survival.

This trial will be the first study to prospectively compare Abraxane-based regimen with a currently standard treatment for squamous histology patients. A total of 120 patients will be randomized at a 1:1 ratio to receive Abraxane 135 mg/m^2^, d1,8 plus carboplatin AUC 5, d1, or gemcitabine 1,250 mg/m^2^ plus carboplatin AUC 5, d1, both in a cycle of three weeks and up to six cycles. The choice of Abraxane dosage and schedule is based on previous researches and the phase III trial result. Weekly Abraxane has been proved to have better efficacy and safety than every three week schedule [13]. Compared to 100 mg/m^2^ d1, 8, 15 in a four-week cycle in the phase III trial, we implement a modified 135 mg/m^2^ , d1, 8 in a three-week cycle schedule to ensure a similar dose intensity but more timely treatment break in order to further reduce toxicity.

The article "A randomized phase II clinical trial of nab-paclitaxel and carboplatin compared with gemcitabine and carboplatin as first-line therapy in locally advanced or metastatic squamous cell carcinoma of lung" was published in 2014. Journal: BMC Cancer.

This study, together with findings from other phase I/II/III studies of Abraxane in NSCLC, will provide valuable insight to the role of Abraxane in the optimal treatment choice for squamous carcinoma of lung.
